# Texture Image Compression Algorithm Based on Self-Organizing Neural Network

**DOI:** 10.1155/2022/4865808

**Published:** 2022-04-10

**Authors:** Jianmin Han

**Affiliations:** School of Computer Engineering, Henan Economic and Trade Vocational College, Zhengzhou, Henan 450046, China

## Abstract

With the rapid development of science and technology, human beings have gradually stepped into a brand-new digital era. Virtual reality technology has brought people an immersive experience. In order to enable users to get a better virtual reality experience, the pictures produced by virtual skillfully must be realistic enough and support users' real-time interaction. So interactive real-time photorealistic rendering becomes the focus of research. Texture mapping is a technology proposed to solve the contradiction between real time and reality. It has been widely studied and used since it was proposed. However, due to limited bandwidth and memory storage, it brings challenges to the stain dyeing of many large texture images, so texture compression is introduced. Texture compression can improve the utilization rate of cache but also greatly reduce the pressure on data transmission caused by the system, which largely solves the problem of real-time rendering of realistic graphics. Due to the particularity of texture image compression, it is necessary to consider not only the quality of texture image after compression ratio and decompression but also whether the algorithm is compatible with mainstream graphics cards. On this basis, we put forward the texture image compression method based on self-organizing mapping, the experiment results show that our method has achieved good results, and it is superior to other methods in most performance indexes.

## 1. Introduction

Due to the limitation of software and hardware of computer system, data compression of digital graphics and images is always the focus of computer graphics research, which has important value in practical application. With the rapid development of science and technology, human beings have gradually stepped into a brand new digital era [1–3]. Digital technology affects every aspect of people's life, among which virtual reality technology has brought people a brand new immersive experience. Its research began in the 1960s. In the early 1990s, it became a relatively complete discipline and aroused great attention. Let users obtain better virtual reality experience; virtual images must have enough sense of reality [3–7]. Therefore, interactive real-time photorealism in virtual reality scenes has become the focus of research. Texture mapping is a technology proposed to solve the contradiction between real time and reality. Texture can obtain realistic details without increasing the complexity of geometric model. Since it was proposed, it has been widely studied and applied [8].

The image has spatial redundancy between adjacent pixels and frequency domain redundancy after DCT. Since the human eye is not sensitive to some signals, the image still has visual redundancy. Removing this redundancy can greatly reduce the storage space required by the image. Image compression technology can reduce the amount of data required for picture preservation and speed up the rate of picture transmission under the premise of keeping the visual quality of pictures basically unchanged. Therefore, image compression has important theoretical and application value and plays an important role in promoting the development of the whole information age [9]. The explosion of mobile Internet users makes many developers transplant applications from PC to mobile terminals. Under the traction of the huge demand for the development of virtual reality, it is imperative for 3D scene visualization to be applied to mobile terminals. However, 3D scene virtual and visualization technology for mobile terminals is still a hot spot and difficulty in current research. Compared with personal desktop computers, mobile terminals of mobile phones have small screen, low resolution, small memory capacity, and limited power [10, 11]. Compared with graphic-based 3D scene visualization methods, the image-based visualization modeling method is suitable for mobile applications due to the low requirements on system hardware capability during rendering and short modeling cycle. For example, texture image data still accounts for 50% to 70% of the massive rendering data. Therefore, massive texture image data still restricts the development of 3D scene visualization in mobile terminals. In order to reduce the amount of texture data transmission, the study of texture image compression technology is extremely urgent [12–14].

Different from general two-dimensional images, texture images contain not only 2D texture color information but also implicit geometry information corresponding to 3D models. Therefore, if geometric information is not taken into account when selecting salient regions, the visually important regions of the texture map cannot be correctly obtained. However, there is no method that considers geometric information in defining the saliency region of texture image. Texture mapping achieves texture image rendering through a large amount of data transmission and calculation, so it puts forward higher requirements on hardware and computing capability of graphic images [15–17]. Texture image rendering is an indispensable key technology to construct 3D scene visualization. After years of development, 3D scene visualization technology has shown great application in the field of application and research. However, even with the rapid development of graphic image hardware and computing capability today [18, 19], the application of 3D scene visualization technology to mobile terminals also needs to overcome the problems of data transmission and computing power consumption [20–24].

This paper consists of five parts. The first and second parts give the research status, background, and related work. The third part is the texture image compression algorithm based on self-organizing neural network. The fourth part shows the experimental results. The experimental results of this paper are introduced and compared and analyzed with relevant comparison algorithms. Finally, the fifth part concludes the full paper.

## 2. Related Work

In the past decades, the field of texture image compression has been widely studied by scholars at home and abroad. This part briefly introduces the origin and development process of texture image compression and gives a brief introduction to some classical texture compression algorithms [25]. Prisma oil painting style change software is available, which uses the Deep Web to transform natural images into art images in the style of oil paintings, which has been downloaded nearly 10 million times in just a few weeks, extending deep learning from science and industry to aesthetics. Image compression is divided into lossy compression and lossless compression. Lossless compression algorithm removes the statistical redundancy of images, and the compression ratio is roughly between 5 : 1 and 2 : 1. Farid et al. [26] proposed a simple format for power image compression, called block clipping coding technique, although it is not in order to solve the texture image compression, but a lot of texture image compression algorithms draw lessons from the idea of it, so that each pixel only needs 2 bits. Ernawan et al. [27] published a paper called “Self-Compressed Texture-Based” in which they listed four texture compression features to illustrate the differences between texture compression and normal image compression methods. Pan et al. [28] used a traditional method called Vector Quantization, or VQ, which compresses the texture image to two or one bit per pixel. However, the vector quantization method, like the palette texture method, requires additional memory access to determine which color to use, which is relatively inefficient, making it unsuitable for the side dyeing pipeline of high performance computer graphic. Penney et al. proposed a new idea fundamentally different from the above method. They obtained two low-resolution texture images from the original texture image and stored them. In the process of decompression, the color of the final texture pixel was obtained by magnifying the two low-resolution images through bilinear interpolation. Armi and Fekri-Ershad [29] concluded advantages and disadvantages of well-known texture image descriptors in the result part. But, the above methods are mainly concerned with recognition performance, computational complexity and antinoise, rotation, etc. A brief review is also made on the common classifiers used for texture image classification.

In the texture compression of wavelet decomposition, Qiao et al. [30] introduced wavelet into the field of texture compression. It is a method of fixed compression ratio proposed based on the energy tightening characteristics of transform. The coefficients of wavelet transform are quantified and then encoded and stored by the standard block compression method. The focus of this approach is to ensure that simple and fast decoding is achieved [31]. The idea is a new one, and it works well. On the same year, this method was formally adopted as an extended standard. Its function is very powerful, supports a range of compression ratios, is basically the most cutting-edge result in the field of texture image compression, but the new method is still to take into account its hardware implementation cost which is relatively high, and is not the most mainstream method, but the future development prospects are very good. With the development of the Internet market, Baidu Map and AutoNavi map have also opened up the market for 3D scene visualization, thus 3D scene visualization has become more and more common into the public's vision, and scholars' research has never been interrupted. Liu et al. [32] proposed to construct procedural syntax, transmit unit texture, and compress redundant texture image data by extracting repeatability and symmetry of 2D texture image. Because the drawing speed is slow three-dimensional scene rendering large amount of calculation, the visualization method based on graphics than most is limited to use desktop for personal desktop, mobile terminal has a small screen resolution, and low memory capacity small data calculation and graphics processing ability is low. Therefore, in the mobile network bandwidth calculation under the premise of limited memory resources, the graphic-based 3D scene visualization method is not suitable for mobile terminal development. In recent years, image-based scene visualization methods have been studied and applied more and more. Some scholars focused on the mosaic and presentation of panoramic images, while some authors study the stretching of panoramic texture images. Deformation and other operations increase the depth of information, but in practical development and application, little attention is paid to the compression of texture image data.

From the above analysis, we know that the above methods have studied the texture image compression widely. However, some problems still exist. For example, no scholar has applied the self-organizing neural network to this field till now, so the research here is still a blank, which has great theoretical research and practical application value for logistics enterprises.

## 3. Texture Image Compression by Self-Organizing Neural Network

### 3.1. Texture Image Compression Process

For example, we tend to draw high level details of characters in movies, such as pore less attention and more attention to the character's facial features. The whole system of the method is given in Figure 1, and the details are as follows: (1) finding the offset threshold; (2) selecting feature points; (3) feature points are iteratively obtained until a satisfactory quantity set is obtained; (4) obtaining texture image feature points 5.

For the progressive grid, not only faces but also edges have tree structure, as shown in Figure 1, because the actual and predicted offset positions of vertices in the grid correspond to each vertex, and each vertex corresponds to an edge in the upper-resolution grid with four edges of one resolution and four edges of the lower-resolution grid Therefore, quadtree of offset can be constructed by constructing quadtree of edge.

### 3.2. Self-Organizing Neural Network

Self-organizing map (SOM) is a neural network that can perform unsupervised learning and clustering of data. Its idea is simple, and it is essentially a neural network with only an input layer and a hidden layer. Armando et al. [33] believed that neurons in different regions of the space had different labor divisions. After the original data are input into the neural network, the network is divided into different response regions according to the response characteristics of each input mode. In the SOM neural network, the mapping relationship between the input layer and the competition layer is shown in the following formula:

(1) $$\begin{array}{c} f:M\Rightarrow N, \end{array}$$

where *M* is the set of input vectors, whose dimension is equal to the dimension of the input vector; *N* varies with the output grid. For example, in the SOM neural network of a two-dimensional grid, N is a two-dimensional plane.

SOM neural network learning algorithm includes three processes: competition, cooperation, and renewal. Competition: the neuron in the network calculates its discriminant function value for each input mode according to the discriminant function, and the neuron with the largest discriminant function value is selected as the winning neuron. Cooperation: the winning neuron influences the spatial location of the excitatory neuron. Update: the excitatory neuron uses its weight adjustment to enhance its response to future similar mode inputs. Calculation of Euclidean distance between weight vector and input vector at mapping layer: at mapping layer, the formula is used to calculate the distance between input sample and each output neuron *J*, as shown in the following formula:

(2) $$\begin{array}{c} d_{j}=\left\|X-W_{j}\right\|=\sqrt{{\sum_{i=1}^{m}\left(x_{i}\left(t\right)-w_{ij}\left(t\right)\right)}^{2}}. \end{array}$$

In the formula, *w*_*ij*_ represents the weight between *i* neuron at the input layer and *j* neuron at the output layer, and the information of all output vectors is stored in each weight vector, that is to say, the weight coefficient represents the relationship between failure symptom and failure mode. The size of input vector and weight vector should keep the same to make the network works.

(3) $$\begin{array}{c} d_{k}=\underset{j}{\min}\left(d_{j}\right). \end{array}$$

The modified formula is shown as follows:

(4) $$\begin{array}{c} w_{ij}\left(t+1\right)=\left\{\begin{array}{cc} w_{ij}\left(t\right)+\eta \left(t\right)\left[x_{i}-w_{ij}\left(t\right)\right], & \left(i\in s_{k}\left(t\right)\right)\text{,}\\ w_{ij}, & \left(i\notin s_{k}\left(t\right)\right)\text{,} \end{array}\right. \end{array}$$

and usually *η*(*t*) to be variational, the details can refer to [33]

(5) $$\begin{array}{c} \eta \left(t\right)=0.2\left(1-\frac{t}{1000}\right), \end{array}$$

or

(6) $$\begin{array}{c} \eta \left(t\right)=\frac{1}{t}. \end{array}$$

We have

(7) $$\begin{array}{c} \sigma_{t}^{2}=\alpha_{0}+\sum_{i=1}^{p}\alpha_{i}\alpha_{t-i}^{2}+\sum_{j=1}^{q}\beta_{j}\sigma_{t-j}^{2}, \end{array}$$

and

(8) $$\begin{array}{c} a_{t}^{2}-\eta_{t}=\alpha_{0}+\sum_{i=1}^{p}\alpha_{i}a_{t-i}^{2}+\sum_{j=1}^{q}\beta_{j}\left(a_{t-j}^{2}-\eta_{t-j}\right). \end{array}$$

So, calculating the output,

(9) $$\begin{array}{c} {Ο}_{k}=f\left(min\left\|X_{j}-W_{j}\right\|\right). \end{array}$$

To ensure that variance is positive, that is, variance exists and is finite [34],

(10) $$\begin{array}{c} \sum_{i=1}^{\max\left(p,q\right)}\left(\alpha_{i}+\beta_{i}\right)<1. \end{array}$$

Once the active node is found, we also want to update neighboring nodes, assigning them an update weight

(11) $$\begin{array}{c} T_{j,I\left(x\right)}=\exp\left(-\frac{S_{j,I\left(x\right)}^{2}}{2\sigma^{2}}\right), \end{array}$$

and then it is time to update the parameters of the node by gradient descent:

(12) $$\begin{array}{c} \Delta w_{ji}=\eta \left(t\right)\cdot T_{j,I\left(x\right)}\left(t\right)\cdot \left(x_{i}-w_{ji}\right). \end{array}$$

(11) updates neighboring nodes and (12) updates the parameters of the node.

A two-dimensional SOM neural network structure is given as Figure 2, which contains the following four parts: (1) array of processing units: receive input signals and form their discriminant functions. (2) Comparison and selection mechanism: compare the discriminant functions and mark the neuron node with the maximum function output value as the winning unit. (3) Local interconnection: when the selected neuron is excited, it will also affect its neighboring neurons. (4) Adaptive process: in this process, the parameters of the excited neuron are constantly modified so that the output value of its discriminant function increases.

## 4. Experimental Results and Analysis

### 4.1. Introduction to Experimental Environment and Data Set

In terms of the selection of data sets, this topic selects Raise and ImageNet data sets as the network training set Raise data set, consisting of 4000 high-resolution and basically lossless images. The Raise data set is composed of 3 different cameras, from Europe 80 multiple locations, including outdoor, indoor, and natural; the size of a picture in a Raise data set is about 4000. 3000 ImageNet data set includes thousands of object categories, and each category contains thousands of pictures.

When the Raise data set is used in this project, all 4000 training images are used to randomly select 50 categories for the ImageNet data set, and then 200 images are randomly selected from these categories to obtain a total of 10000 images from the ImageNet data set. In the process of random selection, images with overexposure and dark size and too small size should be filtered out to avoid a large difference between the image scale exposure of the training set and common natural images.

The hardware environment of the platform was E3-1230 V3 CPU, 32 GB memory, GTX Titan 12 GB video memory, and the PyTorch deep learning framework was used in the Ubuntu 14.04 system experiment. The network uses Adam algorithm to update the gradient and iterates 100 epochs, and the learning rate decayed from 41E in the form of log function.

### 4.2. Experimental Results Analysis

Taken early parameter adjustment: in the process of photo collection, due to the particularity of wide-angle lens, its perspective effect is stronger, edge images are prone to distortion. Therefore, the short focal length lens is not very appropriate in the process of use. As for the choice of focal length, different focal lengths can be selected in different scenes, but one principle must be guaranteed: the pictures are in the same scene. In addition to the shooting angle, all parameters such as focal length, ISO resolution, and aperture speed need to be fixed in order to fix the deformation of the scene and postprocessing, which is shown in Figure 3.

Taken early parameter adjustment: in the process of photo collection, due to the particularity of wide-angle lens, its perspective effect is stronger, edge images are prone to distortion. In addition to the shooting angle, all parameters such as focal length, ISO resolution, and aperture speed need to be fixed in order to fix the deformation of the scene and postprocessing. Postshooting processing: use the PTGui panorama making tool to put all the photos of the same scene into PTGui for processing and output a rough spherical panorama according to the steps of synthesis and adjustment. Then, put the spherical panorama into Krpano and use the batch processing file of Covert SPHERE to CUBE Droplet to form the storage structure of the CUBE panorama model required in this paper.

In this paper, four storage surfaces of cubic panorama are used. According to the principle of scene recognition by the human visual nervous system, the effective area of interest, namely, the area with high complexity, can be quickly recognized according to the scene recognition by the human eye. According to the division of the three levels of areas, each region is divided. The corresponding image resolution is also divided into three levels. The two regions with the largest information entropy, namely, the first level region, are rendered with the highest resolution texture image. The texture image resolution of the two regions in the middle of the order of information entropy size, namely, the second-grade region, is reduced to 0.5 times of the original length and width of the texture image. The length and width of the fingerprint image in Figure 4 were reduced to 0.25 times of the original image in the two regions with the minimum information entropy.

The specific compression effect is shown in Figure 4. Specifically, the image information entropy is used to classify and compress three texture images to achieve multilayer texture image rendering on the same level. This method not only reduces the compression amount of texture data through image scaling but also solves the problem of large computation amount of texture image rendering.

Before using a certain experimental environment and related parameter settings, we give the experimental results of the corresponding database for each encoder, including root mean square error and running time. Besides running time, all values are the average values of all images in the whole database. Red means the method with the shortest running time, and blue means the method with the best quality of decompressed images. For these measures, a smaller RMSE means a smaller error. The higher the PSNR value is, the higher the signal intensity is and the lower the noise is, that is, the better the image quality is. The shorter the run time, the more efficient it is, which is given in Figure 5.

In order to further validate this article, based on the SOM network, a panoramic view of the universal applicability of texture image compression method, the images of acquisition can be divided into two groups, the first set of data is indoor scene and a second group of data is the natural scenery as the main scene (given in Figure 5), and respectively for the two scenarios to experiment, calculate each scene data before and after compression Figure 6.

In scene 1, the total data of texture image in each area before compression is 3511 KB, and after compression, the total data of texture image in each area is 2457 KB, and the compression rate can reach 30.01%. In scene 2, the total amount of texture image data in each area before compression is 3481 KB, and after compression, the total amount of texture image data in each area is 2335.3 KB, and the compression rate can reach 32.91%. The compression rate will be slightly adjusted with different scenes, but the overall compression rate of the scene is above 30%.

The SOM-based panoramic texture image compression method in this paper was used for two different scenes above. From the compression rate, it can be seen that this method is suitable for all different scene compressions, and the compression rate is at least 30%. The 8–12% interest rate range is back in the ascendant. In this experiment, the texture image data is compressed by SOM-based texture image data compression algorithm and compared with the panoramic texture data without this compression method.

It can be seen from Figure 7 that the ICA model can achieve the fastest encoding speed and is better than the fast encoder of some existing DXT1 encoders in terms of quality. The iterative method based on K-means has achieved good results and is faster than the compared algorithms under the condition of similar encoding quality. In addition, increasing the number of iterations can improve the coding quality to a certain extent, but the coding time will increase a lot at the same time. In order to better compare the relationship between measurement indexes of different methods, we gave the line graph corresponding to the operation results of different methods on H databases. Since there are too many methods, it is difficult to draw all indexes on the same graph. We selected the PSNR values that are most used in texture compression quality evaluation for display.

As shown in Figure 8, the *X*-axis represents the original image in the database, and the *Y*-axis represents the ICONS in the PSNR value graph, representing different encoder algorithms. We can see from the figure that our fast coding method Lsq3d achieves good results, which is higher in quality than the other fast modes, and the iterative method based on K-means is in the middle to the upper level of quality. Finally, our combination method achieves the highest PSN values in every image.

As can be seen from the comparative analysis of the above experimental effects. Our method has achieved good results, but there are still shortcomings, especially the quality-oriented method, the image quality obtained by this method is as good as the existing best DXT1. There are still some gaps in the encoder, so we use the combination method, which beats all the encoders in quality, but the encoding time is much slower, and our combination method has no significant improvement in quality compared with other methods.

As shown in Figure 9, when the K-means algorithm is applied to the set of image feature points, the selection of the initial number of seed points needs to be discussed. First, the number of seed points determines the number of classes after the aggregation of feature points. A larger number of seed points can be used to generate a larger number of classes, which will ensure the accuracy of the ROI region extracted because each class occupies too small area, and too few seed points will cause the number of classes. Each class covers the area of the zone too interested in the results of the accuracy which is not high. Second, because of the information on the 3*D* model surface, the surface feature points do not reflect the importance of surface area. Only the set of feature points were distributed in the middle of the area, this area can be seen as area of interest, and after three-dimensional space to two-dimensional space mapping, some feature points in the UV coordinates are coincidence points; the overlap will affect the result of the experiment, need to be removed. Experiments have shown that an initial number of 300 seed points is usually appropriate.

## 5. Conclusions

Most of the information people get from the surrounding environment comes from vision, and the study of visual images has always been an important direction in the field of scientific research. After entering the information age, people's demand for the quality of digital pictures is getting higher and higher, so digital pictures are developing towards clearer and higher resolution methods to increase the amount of picture data. In recent years, the growth rate of image data exceeds the technological development of storage and transmission speed. It is unrealistic to rely on increasing storage capacity and network bandwidth. We can only consider the image content itself and design image compression algorithm reasonably. When the visual distortion of the image is small, the redundant information of the image should be removed as much as possible to reduce the consumption of storage and bandwidth.

Neural network model can fully excavate the essential information of the image and separate the important features and unimportant redundant information in the image and has a strong potential in the field of image compression. This topic uses deep convolutional network to deal with the problem of image codec, so that the image has a better compression effect. Although the method in this paper aims at the image-based cubic panoramic texture image data, however, the spherical and cylindrical panoramic texture image data can also have a good application in the field of graphic image-based modeling, which provides a new idea for efficient rendering of texture image in 3D scene visualization. The application of the new method in spherical and cylindrical panoramic modeling will be further studied. For deep learning processing of image compression, there are still many aspects to be further studied, such as entropy rate control module in full roll machine network coding and image quality evaluation criteria when using adversarial network.

## Figures and Tables

**Figure 1:** The image compression diagram of SOM networks.

**Figure 2:** Two-dimensional SOM neural network structure.

**Figure 3:** Take samples of adjacent photos.

**Figure 4:** Compression result of fingerprint image.

**Figure 5:** Data compression ratio results of different data sets.

**Figure 6:** A display of the two scenarios.

**Figure 7:** Image compression results display based on SOM.

**Figure 8:** The results of compressed SNR by different methods.

**Figure 9:** Compression results of physical images at different angles.

## Data Availability

The data used to support the findings of this study are available from the author upon request.
